# Analysis of Cosmetic Effect of Nanocomposite Resin on Anterior Teeth

**DOI:** 10.1155/2021/7367320

**Published:** 2021-11-30

**Authors:** Yubo Wang, Junfu Li, Daiyun Chen, Li Li

**Affiliations:** ^1^Department of Prosthodontics, Qingdao Stomatological Hospital Affiliated to Qingdao University, Qingdao, China; ^2^Department of Stomatology, The Second Affiliated Hospital of Shandong First University, Shandong, China; ^3^Department of Pediatric Dentistry, Qingdao Stomatological Hospital Affiliated to Qingdao University, Qingdao, China

## Abstract

The problems of anterior teeth include dental plaque, dental caries, and fracture, which are usually treated with common composite resin clinically. Although good repair effect can be achieved, patients are prone to anterior tooth sensitivity after surgery. Therefore, the purpose of this study is to analyze the cosmetic effect of nanocomposite resin on anterior teeth. Up to 176 patients (176 teeth) undergoing anterior dental cosmetic restoration in our hospital were selected and assigned to the LR group (*n* = 88) and the NR group (*n* = 88) according to patients' voluntary choice of prosthetic materials. The LR group was cured with light-cured composite resin, while the NR group was cured with nanocomposite resin. By comparing the related indexes of patients in the two groups, it was discovered that in the NR group, the excellent and good rate and patients' evaluation of the repair effect were higher, while the periodontal attachment, gingival index, dental plaque index, VAS score, and the incidence of tooth sensitivity were lower, all *P* < 0.05. The results indicated that the nanocomposite resin had significant cosmetic effect on anterior teeth and had application value.

## 1. Introduction

There are 12 anterior teeth, including single canines, central incisors, and lateral incisors, which have chewing, pronunciation, and aesthetic functions [1]. Trauma caused by a variety of reasons can cause anterior tooth caries, fracture, dental plaque, and other problems, which not only lead to poor appearance of patients but also affect the normal life. Therefore, there is an urgent need for anterior tooth cosmetic restoration, and the requirements for the restoration effect are also increasing day by day. They require not only the firm and reliable restoration of teeth but also the aesthetic appearance of teeth [2]. In clinical practice, the focus of dental restoration is placed on the problems of prosthesis and gingival [3]. Anterior tooth restoration is aimed at realistic and healthy teeth as well as beautiful gingival tissue. It systematically trigs the color, shape, and arrangement direction of anterior teeth, which combines technical and aesthetic contents [4]. Different dental restorative materials have different restorative effects on occlusal function, edge fit, color, shape, and incidence of complications [5]. At present, light-cured composite resin is widely used in tooth repair. Under ultraviolet irradiation, it is polymerized by photosensitizer and can be highly bonded to teeth. In addition, it can also fill a large area of deep caries and has the characteristics of accurate molding, vivid color, and easy operation [6]. However, the teeth repaired with light-cured composite resin materials are easy to fall off and become sensitive, thus affecting the function of the anterior teeth. Therefore, it is of positive significance to explore a kind of beautiful and stable anterior restorative material for patients. Filtek Z350 nanocomposite is a new type of curing composite material with hard texture and color of dentin, tooth body, tooth enamel, and transparent. These colors are very similar to the tooth body color and can perfectly combine the durability and polish of teeth [7]. However, there are few reports on the application of Filtek Z350 nanocomposite resin in anterior tooth restoration, so it is necessary to explore the effect of nanocomposite resin on anterior tooth restoration. The purpose of this study is to analyze the cosmetic effect of nanocomposite resin on anterior teeth and provide data reference for clinical practice. The results were reported as follows.

## 2. Materials and Methods

### 2.1. Patients' Information

After the approval of the Medical Ethics Committee, the patients who underwent anterior dental cosmetic restoration in our hospital from July 2018 to July 2020 were selected as the research objects. Inclusion criteria were as follows: (1) defect of anterior teeth was determined upon admission [8]; (2) local moisture separation of teeth can be performed [9]; (3) they were able to communicate in normal language; (4) there was no coagulation dysfunction. Exclusion criteria are as follows: (1) need to bear large bite force; (2) complicated mental diseases; (3) complicated with organic diseases of the heart, liver, kidney, and other important organs; and (4) women in pregnancy or lactation. In the end, up to 176 patients (176 teeth) were elected and split into the NR group and the LR group with 88 cases each according to patients' voluntary choice of prosthetic materials. Comparison of gender, age, and anterior tooth defect causes between the two groups showed *P* > 0.05, indicating no significant difference and having comparability (Table 1).

### 2.2. Anterior Dental Cosmetic Restoration Method

The research method flow is shown in Figure 1. Primary treatment of anterior teeth: in the early stage of repair, the tooth defect was examined in both groups, followed by tooth surface cleaning, decaying material removal, and tooth body and necrotic tissue grinding. For the patients with decayed anterior teeth, the defects were repaired and fixed according to the cavity shape after retaining healthy teeth. For patients with obvious wide dental space, 3M self-etching binder was given for etching treatment and then repair. For patients with incomplete tooth enamel, the tooth enamel should be removed and the restoration procedure should be performed. Anterior tooth retreatment: patients in both groups were treated with 3M self-etching binder for 30 seconds, light curing for 20 seconds, and colorimetry (after colorimetry under natural light, a material similar in color to the patient's front teeth was selected). Anterior tooth restoration: the anterior teeth of the LR group were repaired with light-cured composite resin (Filtek Z100), and the anterior teeth of the NR group were repaired with nanocomposite resin (Filtek Z350) (Figure 2). Both materials were provided by 3M China Co., Ltd. Each layer of the filling material was cured for 40 seconds, and then, the patient's front teeth were grinded and polished by using polishing paste, throwing optical discs, and polishing strips in the principle of from coarse to fine. Instruction client was to grind and polish properly after occlusion to ensure that the front teeth were in perfect alignment with the lower teeth and the surrounding teeth.

### 2.3. Observation Indicators

The restoration effect: after the restoration treatment, the restoration effect of the patient's anterior teeth was evaluated. Excellent: the occlusal function of the anterior teeth returned to normal. The edge fit was good. The color and appearance were beautiful, and there were no complications. Good: the occlusal function of the front teeth is basically restored. The edge fit, color, and shape are normal or slightly defective, no complications. Bad: not up to a good and excellent standard. Excellent and good rate = (excellent + good) case number/total case number × 100% [10].

Periodontal health status: the community periodontal index (CPI) was used to check the periodontal health status of patients [11]. The examination method was to use CPI probe combined with visual examination. The examination areas were the left upper posterior dental area, the left lower posterior dental area, the right upper posterior dental area, the right lower posterior dental area, the anterior dental area, and the lower anterior dental area of index teeth. The examination items were calculus, periodontal pocket depth, and gingival bleeding. Hold the CPI probe in pen style and slowly insert it into the periodontal pocket so that the probe was parallel to the tooth axis and attached to the root of the tooth. By moving the CPI probe far and near along the labial and lingual gingival crevices of the teeth, the subgingival stones (calculus examination) were felt and the gingival bleeding was checked at the same time. The scale of the CPI probe is the periodontal pocket depth (periodontal pocket depth examination). Note that the CPI probe should be used with a force of less than or equal to 20 g. The score is shown in Table 2.

Pain scale: Visual Analogue Scale (VAS) was used to assess patients' pain at 4, 8, and 12 weeks after repair [12]. Detection method: scale values of 0-10 cm scale plate were used to represent different degrees of pain. Patients were allowed to feel the pain by themselves and marked on the scale to represent the degree of pain. 0 points meant painless and 10 points meant severe pain.

The satisfaction rating of patients on the effect of anterior tooth restoration: the satisfaction questionnaire made by our hospital was used to evaluate the patients on the four aspects of psychology, facial appearance, tooth appearance, and tooth color. The full score of each item was 100, and the higher the score was, the more satisfied the patients were. Incidence of tooth sensitivity: patients were observed for tooth sensitivity within 4 weeks after restoration and recorded. Criterion for judging tooth sensitivity: when a tooth was stimulated by cold, hot, sour, or sweet or when a tooth is rubbed or bitten hard, it may produce transient or temporary persistent pain symptoms, and the pain will disappear when the stimulation ends [13].

### 2.4. Data Statistics

SPSS 20.0 statistical software was adopted. Qualitative data were expressed by percentage, carrying out the chi-square test. When comparing the data with theoretical frequency of 1 to 4, the chi-square should be corrected. Quantitative data were represented as median, performing *t*-test. Repeated measurement analysis of variance was used to compare data at multiple time points. *P* < 0.05 was deemed statistically significant.

## 3. Results and Discussion

### 3.1. Repair Effect and CPI

Compared to that of the LR group, the excellent and good rate of the NR group was higher (96.59% vs. 85.23%) (Table 3, Figure 3). In addition, the periodontal attachment, gingival index, and dental plaque index were lower (Table 4, Figure 4). The *P* for all comparisons were <0.05.

### 3.2. VAS Score and Patients' Evaluation of the Repair Effect

The VAS score decreased with time in both groups, and the NR group manifested lower, with an interaction effect between the groups and time (between-group effect: *F* = 1231.000, time effect: *F* = 1167.000, interaction effect: *F* = 122.500, all *P* < 0.001) (Table 5, Figure 5).

### 3.3. The Score of the Patients on the Restoration Effect and the Incidence of Tooth Sensitivity

The scores of psychology, facial features, tooth appearance, and tooth color in the NR group were higher (*P* < 0.05) (Table 6, Figure 6). Dental sensitivity was observed in 9 patients (10.23%, 9/88) of the NR group and 26 patients (29.55%, 26/88) of the LR group (*χ*^2^ = 10.307, *P* = 0.001) (Figure 7).

## 4. Discussion

In response to people's needs, anterior restorations should be both beautiful and durable. The common photocurable composite resin has obvious shrinkage, weak wear resistance, and low mechanical strength, which leads to some problems such as falling off and cracking after it is applied to tooth repair [14]. Nanocomposite resin is a category of nanomaterials. It is made up of smaller than 100 nm of crystalline and amorphous structure units, with special structural characteristics and performance and can show excellent performance. It provides a new direction for the front tooth repair material selection. So the nanocomposite resin has the vital significance of the effects of anterior tooth restoration.

In this study, the excellent and good rate and scores of psychological, facial appearance, tooth appearance, and tooth color of patients treated with nanocomposite resin materials were significantly higher than those of patients treated with light-cured composite resin materials, indicating that these patients had better repair results. The reason may be that the Z350 nanocomposite resin selected by the patient is translucent and has excellent shading performance, which is very similar to the original color of the patient's defective tooth without discoloration or coloring [15]. In addition, the contact area between the nanosized particles contained in the Z350 nanoresin and the group after silane treatment increases greatly, which weakens the polymerization shrinkage of the resin. As a result, the composition of the nanoresin increases, and the polishing property and polishing retention are also enhanced [16]. Therefore, it can ensure smooth surface and complete appearance and beautiful appearance after bonding the defect tooth surface. Edge closeness is a factor to evaluate whether the restoration can function normally for a long time. The higher the edge closeness is, the higher the flexural strength is. And the less prone the tooth is to crack after restoration, the longer the tooth can be used [17]. The resin shrinkage of Z350 nanocomposite resin can make the filling contact with the tooth tissue more fully and closely and improve the edge fit. In addition, Z350 nanocomposite resin combines the advantages of ordinary composite resin (such as simple operation, natural color, accurate plasticity, suitable flow, and wear resistance) and nanocharacteristics. The gap between nanoscale particles in the packing is very small, which makes it difficult for bacteria and water in the oral cavity to enter and damage the dental pulp, reducing complications such as gingivitis and secondary caries, ensuring the vitality of the dental pulp, improving the occlusal function of the anterior teeth [18]. Therefore, the restoration effect of Z350 nanocomposite resin is significant, which makes patients' psychological, facial appearance, tooth appearance, tooth color, and other aspects better evaluated after restoration, which is similar to the results of relevant studies [19]. In this study, all patients were examined by CPI, and it was found that the periodontal attachment, gingival index, and dental plaque index of the patients treated with nanocomposite resin materials were significantly reduced, indicating that these patients had healthier periodontal tissues [20]. CPI is easy to operate and has good repeatability. It is widely used in the examination of periodontal health. The low VAS score of patients treated with nanocomposite resin material after restoration indicates that nanocomposite resin material can reduce the pain of patients with restoration, which may be related to the reduction of dental neuroinflammation in patients [21]. The results of this study showed that the use of nanocomposite resins significantly reduced the incidence of tooth sensitivity. The reason may be that Z350 nanocomposite resin has strong compression resistance, polishing property, and edge suitability. Nanosized particles have very small diameter and can enter the polymer chain gap, so the probability of dental pulp stimulation is very low, which effectively reduces the occurrence of tooth sensitivity after restoration [22]. The sample size of this study is limited, and further confirmation is needed with a larger sample size.

## 5. Conclusion

Z350 nanocomposite resin belongs to the composite superfine packing resin, by nanoscale (within 100 nm) particles and group, after the silane treatment greatly increasing the contact area. So it can avoid the polymerization and contraction of the resin so that the filling material and the tooth tissue close and full contact. Moreover, it has strong solidification adhesion with tooth tissue, reducing tooth wear, and has durability, tensile resistance, and compression resistance. Compared with the light-cured composite resin material, the nanocomposite resin material had a higher excellent and good rate and healthier periodontal tissue for the repair of anterior tooth caries, wide tooth space, and incomplete tooth enamel. Patients felt less pain and were more satisfied with the repair effect, which was worthy of application.

## Figures and Tables

**Figure 1:** Experimental process. Patients requiring cosmetic restoration of anterior teeth were selected and split into groups. The LR group was cured with light-cured composite resin material, while the NR group was cured with nanocomposite resin material. The related indexes of the two groups were compared.

**Figure 2:** Nanocomposite resin. (a) Z350 nanocomposite resin. Z350 nanocomposite resin is used in the cosmetic restoration of anterior teeth, which has little pulling force on tooth tissue. (b) Electron microscopy of Z350 nanocomposite resin. The Z350 nanocomposite resin particles are round under an electron microscope.

**Figure 3:** Repair effect. The excellent and good rate of the NR group was significantly higher, *P* < 0.05.

**Figure 4:** Community periodontal index (CPI). Periodontal attachment, gingival index, and dental plaque index in the NR group were all lower, *P* < 0.05.

**Figure 5:** Visual Analogue Scale (VAS). The VAS score of the NR group was lower, *P* < 0.05.

**Figure 6:** Repair effect score. The scores of mentality, facial features, tooth look, and tooth color in the NR group were higher, *P* < 0.05.

**Figure 7:** The occurrence of tooth sensitivity. The incidence of tooth sensitivity in the NR group was lower (10.23% vs. 29.55%), *P* < 0.05.

**Table 1:** Patient's gender and anterior tooth defect causes.

Group	Gender (case)		Gender (*x̅*±*s*, year)	Anterior tooth defect causes (case)			
	Male	Female		Fluorotic teeth	Injury	Wedge shape	Decayed tooth
LR group (*n* = 88)	41 (46.59%)	47 (53.41%)	50.04 ± 4.27	12 (13.64%)	13 (14.77%)	8 (9.09%)	55 (62.50%)
NR group (*n* = 88)	39 (44.32%)	49 (55.68%)	49.58 ± 4.03	10 (11.36%)	7 (7.95%)	11 (12.50%)	60 (68.18%)
*χ* ^2^/*t*/*Z*	0.092		0.735	-0.932			
*P*	0.762		0.463	0.352			

**Table 2:** CPI score situation.

Score	Representative
0	Healthy gums.
1	This is gingivitis, which may present as postexploratory bleeding.
2	Tooth stone, the manifestation of the exploration can be seen calculus.
3	In early periodontal disease, the gingival margin covered part of the black part of the probe, and the depth of the periodontal pocket was 4–5 mm.
4	In advanced periodontal disease, the gingival margin completely covered the black part of the probe, and the depth of the periodontal pocket was more than 6 mm.
X	Excluded section (less than 2 functional teeth).
9	Unable to check.

**Table 3:** Repair effect.

Group	Number of repaired teeth	Bad	Good	Excellent	Good + excellent
LR group	88	13 (14.77%)	35 (39.77%)	40 (45.45%)	75 (85.23%)
NR group	88	3 (3.41%)	40 (45.45%)	45 (51.14%)	85 (96.59%)
*t*					5.569
*P*					0.018

**Table 4:** CPI (*x* ± *s*, point).

Group	Number of repaired teeth	Periodontal attachment	Gingival index	Dental plaque index
LR group	88	2.41 ± 0.75	2.03 ± 0.61	1.32 ± 0.32
NR group	88	1.86 ± 0.84	1.55 ± 0.49	1.08 ± 0.17
*t*		4.582	5.755	6.213
*P*		<0.001	<0.001	<0.001

Note. CPI: community periodontal index.

**Table 5:** VAS score (*x* ± *s*, point).

Time	LR group (*n* = 88)	NR group (*n* = 88)	*t*	*P*
Before repair	7.58 ± 0.95	7.41 ± 1.34	0.971	0.333
4 weeks after repair	5.76 ± 1.18	2.16 ± 0.41	27.030	<0.001
8 weeks after repair	4.35 ± 0.87	1.17 ± 0.35	31.810	<0.001
12 weeks after repair	3.27 ± 1.21	0.77 ± 0.36	18.580	<0.001

Note. VAS: Visual Analogue Scale.

**Table 6:** Repair effect score (*x* ± *s*, point).

Group	Mentality	Facial features	Tooth look	Tooth color
LR group (*n* = 88)	90.16 ± 14.63	83.95 ± 15.26	84.22 ± 14.39	85.66 ± 13.58
NR group (*n* = 88)	95.57 ± 17.12	96.21 ± 16.13	93.84 ± 15.58	95.19 ± 16.28
*t*	2.254	5.180	4.255	4.217
*P*	0.025	<0.001	<0.001	<0.001

## Data Availability

All the raw data could be accessed by contacting the corresponding author for any qualified researcher need.
